# Can the addition of radiotherapy postoperatively increase clinical outcome of patients with gastric cancer? A systematic review of the literature and meta-analysis

**DOI:** 10.18632/oncotarget.23754

**Published:** 2017-12-28

**Authors:** Francesco Fiorica, Marco Trovò, Alessandro Ottaiano, Guglielmo Nasti, Ilaria Carandina, Marina Marzola, Paolo De Paoli, Massimiliano Berretta

**Affiliations:** ^1^ Department of Radiation Oncology, University Hospital Ferrara, Ferrara, Italy; ^2^ Radiotherapy Division, “Santa Maria della Misericordia” Hospital Udine, Udine, Italy; ^3^ Division of Abdominal Medical Oncology, National Cancer Institute, “Pascale” Naples, Naples, Italy; ^4^ Department of Medical Oncology, University Hospital Ferrara, Ferrara, Italy; ^5^ Scientific Directorate, National Cancer Institute (CRO), Aviano (PN), Italy; ^6^ Division of Medical Oncology A, National Cancer Institute (CRO), Aviano (PN), Italy

**Keywords:** radiotherpy gastric cancer, adjuvant therapy gastric cancer, radiochemotherapy gastric cancer

## Abstract

**Background:**

Although several studies have been carried out to determine the best treatment for gastric carcinoma, the data on survival rate still remain inconclusive.

**Objective:**

To evaluate the effects of postoperative radio-chemotherapy on overall and disease-free survival.

**Data Sources:**

MEDLINE and CANCERLIT searches of reference lists (for the period 1970 to 2016) were supplemented with hand search of reference lists.

**Study selection:**

The present work includes randomized controlled trials comparing postoperative radio-chemotherapy to postoperative chemotherapy or to surgery alone in patients with resected gastric carcinoma without evidence of metastatic disease. Ten randomized controlled trials were analyzed in total: four compared postoperative radiochemotherapy to surgery alone (708 patients), and six compared postoperative radiochemotherapy to postoperative chemotherapy (1020 patients).

**Data extraction:**

According to “intention to treat” method, three independent observers have extracted from each trial, the data on patients, intervention, and outcomes. These data were subsequently combined using DerSimonian and Laird methods.

**Results:**

Postoperative radiochemotherapy significantly increases 3-year and 5-year overall survival and 3-year and 5-year disease free survival rate compared to postoperative chemotherapy (RR 0.89; 95%CI 0.81-0.97 and RR 0.82; 95%CI 0.71–0.95) or surgery alone (RR 0.83; 95% CI 0.77-0.91 and RR 0.80; 95% CI 0.65–0.98).

**Conclusions:**

In patients with resected gastric cancer, postoperative radiochemotherapy obtains: 1) an increase in overall survival, 2) an increase in disease free survival, and 3) a gain in 5 year disease free survival independent of surgical procedure.

## INTRODUCTION

Gastric carcinoma continues to represent an enigmatic and heterogeneous disease [1] also for its management. Gastric cancer is the fifth most common cancer in the world: despite significant improvements, it still is the third cause of death among cancer patients [2]. In 2007, a pooled analysis [3] of randomized clinical trials, including the Gastric Surgical Adjuvant Trial (INT0116) [4], showed that radiotherapy (RT) significantly increases 3-year and 5-year overall survival:even though the improvement is relatively limited it still is clinically important.

Performed along with adjuvant studies, the MAGIC trial demonstrate the advantage of preoperative chemotherapy, thus becoming the standard of treatment. [5] Furthermore, improvements in surgical technique showed an important role of lymphadenectomy to tumor stage accurately and to increase long-term survival. In Europe, a gastrectomy with dissection of perigastric nodes and second echelon lymph-nodes, the so-called D2 resection (at least 16 nodes for pathologic evaluation) is considered standard in curative-intent surgery [6]. In advanced gastric cancer, several studies have evaluated the impact of “super-extended” lymphadenectomy (D3 resection) on recurrences, suggesting that it does not decrease locoregional recurrences [7].

That being so, about 50% of advanced gastric cancer patients will experience a recurrence, more specifically about 30% will experience local recurrence. [8]. This high risk of recurrences, even when resection has been considered curative, makes advanced gastric cancer a hardly curable disease, although still treatable. Even if a standardized surgery with lymphadenectomy was used, radiochemotherapy combined with surgery could increase disease control. Since the results of randomized studies are inconsistent, it is hard to gauge the effect of combined treatment on survival. However, improved survival remains the main goal in the management of advanced gastric cancer.

The objective of this meta-analysis and systematic review were to provide a comprehensive and reliable summary of adjuvant radiation therapy effects regarding 3-year and 5-year overall survival and 3 year and 5 year disease-free survival and to examine and interpret heterogeneity in results.

### Characteristics of the RCTs

The bibliographic search retrieved 123 studies of which ten respected the inclusion criteria and were therefore included. After excluding the studies without inclusion criteria, ten RCTs were included [14, 15, 16, 4, 17, 18, 19, 20, 21, 22]. The study selection procedure is presented in Figure 1. In this meta-analysis randomized clinical trials evaluating the addition of postoperative radiotherapy to surgery only and surgery and adjuvant chemotherapy, treating patients without metastatic disease and with a resected histologically proven gastric carcinoma, and having overall survival as an outcome measure of the effect of the treatment were included. Two reviewers (F.F. and M.M.) blindly decided which study was to be included, any disagreements were overcome discussing. Excluded RCTs were related to the purpose behind avoidance. Excluded studies were non-randomized or published as a preliminary report and later published as a final paper. If more than one publication reported the results of a same study, only the publication with the latest and full data were included in the meta-analysis. [23]. A trial [24] was excluded due to its use of a very different chemotherapeutic schedule (doxorubicin added to 5-fluorouracil and methyl-CCNU)as part of a combined treatment. The major characteristics of trials included in the meta-analysis are presented in Table 1.

**Figure 1:** Flowchart of the literature search and selection process

**Table 1:** Patient characteristics in trials included in the meta-analysis

Study [reference]	Year	Treatment arm	Sample size (n)	Male (%)	Mean Age	Performance (%)		Location of primary (%)		*N* Stage (%)		Stage (%)		Surgical procedures (%)			Linfoadenectomy procedures
						≤ 1	>1	Cardias	Corpus/Antrum	N0	N+	< III	≥ III	Total gastrectomy	Partial gastrectomy	others	
Dent et al. [14]	1979	S+CRT S	35 31	n.r. n.r	n.r. n.r.	n.r. n.r.	n.r. n.r.	n.r. n.r.	n.r. n.r.	37 29	63 71	n.r. n.r.	n.r. n.r.	Not specifed	Not specifed	Not specifed	Not specifed
GTSG [15]	1982	S+CRT	45	73	n.r.	64	36	24	76	n.r.	n.r.	n.r.	n.r.	Not specifed	Not specifed	Not specifed	Not specifed
		S+CT	45	67	n.r.	76	24	20	80	n.r.	n.r.	n.r.	n.r.				
Moertel et al. [16]	1984	S+CRT	39	74	58	n.r.	n.r.	49	51	18	82	n.r.	n.r.	10	17	0	Not specifed
		S	23	74	56	n.r.	n.r.	56	44	22	78	n.r.	n.r.	90	83	0	
MacDonald et al. [4]	2001	S+CRT	281	72	60	94	6	21	79	14	86	n.r.	n.r.	Not specifed	Not specifed	Not specifed	D0 resection: 54% D1 resection: 36% D2 resection: 10%
		S	275	71	59	94	6	18	82	16	84	n.r.	n.r.				
Kwon et al. [18]	2010	S+CRT	31	68	56	100	0	20	80	n.r.	n.r.	0	100	Not specifed	Not specifed	Not specifed	D2 resection: 100%
		S+CT	30	77	49	100	0	13	87	n.r.	n.r.	0	100				
Bamias et al. [17]	2010	S+CRT	72	67	55,8	99	1	20	80	22	78	25	75	39	49	12	D0 resection: 56% D1-2 resection: 44%
		S+CT	71	73	56,1	99	1	26	74	15	85	32	67	41	53	6	
Yu et al. [20]	2012	S+CRT	34	65	54	30	70	20	80	0	100	0	100	32.2	35.6	32.2	D1 resection: 34% D2 resection: 66%
		S+CT	34	62	55	26	74	26	74	0	100	0	100	30.2	41.5	28.3	
Kim et al. [19].	2012	S+CRT	46	74	54.5	n.r.	n.r.	51	49	49	51	0	100	35.1	32	32.9	D2 resection: 100%
		S+CT	44	57		n.r.	n.r.	35	65	45	55	0	100	26.7	41.3	32	
Zhu et al. [21]	2012	S+CRT	186	72.9	59	100	0	9.9	90.1	13.3	86.7	30.2	69.8	Not specifed	Not specifed	Not specifed	D2 resection: 100%
		S+CT	165	76.4		100	0	16.1	83.9	15.1	84.9	27.3	72.7				
ARTIST [22]	2015	S+CRT S+CT	230 228	62.2 67.1	56	42 43	58 57	6 4	85 87	12 15	88 85	42 41	58 59	Not specifed	Not specifed	Not specifed	D2 resection: 100%

In total, the 10 RCTs [14, 15, 16, 4, 17, 18, 19, 20, 21, 22] included 1944 patients, 997 of whom received radiotherapy combined with chemotherapy.

Inclusion criteria were uniform in all but one RCT, which included only resectable patients with a poor prognosis [16]. Four studies [15, 4, 21, 22] were multicenter. There were a great variability in the sample size of each RCT, ranging from 30 [18] to 281 [4] patients. The rate of males ranged from 58% [19] to 76.4% [21]. Mean age was 56 years, ranging from 49 [18] to 60 years [4].

Table 1 reports data on surgical technique employed, and the rate of resection (curative or palliative). In six trials [4, 18, 19, 20, 21, 22], the rate of D0 versus D1 versus D2 resection was described. In all trials, resection was defined as “curative” when margins of the resected tissue were regarded “free of tumor” by both surgeon and pathologist, in agreement. There was a great variability in proportion of patients with a curative resection in all trials ranging from 0% to 100%. The rates of patients with positive nodes and stage III and IV varied in RCTs (ranging from 63% to 88% and from 59% to 100%, respectively). In three RCTs [15, 21, 22] the method of randomization was not adequately described. In none of these studies an adequate treatment allocation concealment was used: it was therefore impossible to perform blinding due to the nature of radiochemotherapy trials.

### Source of support

This meta-analysis was totally sustained by the authors’ institutions.

## RESULTS

### 3- and 5-Year overall survival

The effect of adding radiotherapy to postoperative chemotherapy or to surgery alone on 3-year overall survival (8 RCTs: 1793 patients, 980 alive subjects) is reported in Figure 2. The addition of RT enhanced overall survival in the postoperative setting in all RCTs. However, a statistically significant difference was found in only one case [4]. The range of RR in each trial was comprised between 0.58 and 1.06. The pooled estimate of the treatment effect was significant (RR 0.89 (95% CI 0.81–0.97); *p* = 0.01) (NNT = 17). Comparable results were acquired when a fixed-effects model was used (RR 0.87 (95% CI 0.79–0.96); *p* = 0.004). With “robust analysis” excluding one study at a time and therefore - evaluating 8 RCTs, a lost statistical significance for 3-year overall survival omitting the trial by MacDonald was demonstrated [4].

**Figure 2:** 3-year overall survival Meta-analysis of eight RCTs of radiochemotherapy: four RCTs of postoperative radiochemotherapy vs. postoperative chemotherapy (**A**), four RCTs of postoperative radiochemotherapy vs. surgery alone (**B**). The relative risk (RR) and 95% confidence interval (CI) for the effect of treatment on 3-year overall survival are shown on a logarithmic scale. Studies are arranged by publication year.

Five-year survival was reported in 8 RCTs (1811 patients: 877 alive subjects). Figure 3 shows the benefit of postoperative radiochemotherapy on 5-year overall survival. In all RCTs, radiation added postoperatively increased the survival, however a significant benefit was observed in one trial only [4]. The RR range was between 0.77 to 1.01. The pooled estimate of the treatment effect was significant (RR 0.83, 95% CI 0.77–0.91); *P* < 0.00001) (NNT = 11). Comparable results were acquired when a fixed-effects model was used (RR 0.83, 95% CI 0.77–0.91); *p* < 0.00001). This impact on 5-year overall survival was found not to be related to any RCT.

**Figure 3:** 5-year overall survival Meta-analysis of eight RCTs of radiochemotherapy: five RCTs of postoperative radiochemotherapy vs. postoperative chemotherapy (**A**), 3 RCTs of postoperative radiochemotherapy vs. surgery alone (**B**). The relative risk (RR) and 95% confidence interval (CI) for the effect of treatment on 5-year overall survival are shown on a logarithmic scale. Studies are arranged by publication year.

### 3- and 5-Year disease-free survival

The effect of adding radiotherapy to surgery or to adjuvant chemotherapy on 3-year disease-free survival (7 RCTs: 1789 subjects, 1130 patients without recurrences) is reported in Figure 4. The pooled estimate of the treatment effect on 3-year disease-free survival was significant (RR 0.81 [95% CI, 0.72–0.92] p=0.0007) (NNT = 14). Comparable results were acquired when a fixed-effect model was used.

**Figure 4:** 3-year disease free survival Meta-analysis of eight RCTs of radiochemotherapy: six RCTs of postoperative radiochemotherapy vs. postoperative chemotherapy (**A**), two RCTs of postoperative radiochemotherapy vs. surgery alone (**B**). The relative risk (RR) and 95% confidence interval (CI) for the effect of treatment on 3-year disease free survival are shown on a logarithmic scale. Studies are arranged by publication year.

Furthermore, the effect of the addition of radiotherapy on 5-year disease-free survival (7 RCTs: 1721 patients, 885 subjects without recurrences) is presented in Figure 5. The addition of radiotherapy favored 5-year disease-free survival in all RCTs but one [17], however a statistically significant benefit was observed in only one RCT [4]. The RR range in each trial was between 0.56 to 1.04. The pooled estimate of the treatment effect was significant (RR 0.80 [95% CI 0.72–0.89]; *p* < 0.0001) (NNT = 9). Comparable results were acquired with a fixed-effects model (RR 0.79 [95% CI 0.72–0.876]; *p* < 0.00001). With “robust analyses”, no significant differences in treatment effect estimate were reported.

**Figure 5:** 5-year disease free survival Meta-analysis of seven RCTs of radiochemotherapy: five RCTs of postoperative radiochemotherapy vs. postoperative chemotherapy (**A**), two RCTs of postoperative radiochemotherapy vs. surgery alone (**B**). The relative risk (RR) and 95% confidence interval (CI) for the effect of treatment on 5-year disease free survival are shown on a logarithmic scale. Studies are arranged by publication year.

### Postoperative radiochemotherapy versus Postoperative chemotherapy

Four RCTs (1020 patients) on the postoperative addition of radiotherapy to chemotherapy vs. postoperative chemotherapy were combined in this 3-year overall survival analysis [17, 20, 21, 22]; 521 patients were treated with postoperative radiochemotherapy and 499 with postoperative chemotherapy. A significant benefit in 3-year overall survival (RR 0.83 [95% CI 0.70–0.98]; *p* = 0.03), NNT = 14 (Figure 2A) was revealed when pooling the data from these four studies. Evaluating 5-year outcome, no difference in overall survival was demonstrated (RR 0.89 [95% CI 0.77–1.02]; *p* = 0.09) (Figure 3A).

The effect of postoperative radiochemotherapy on 3-year disease-free survival (5 RCTs [17, 18, 20, 21, 22] : 1789 patients, 1130 subjects without disease recurrence) is shown in Figure 4A. The pooled estimate of the treatment effect was significant (RR 0.82 [95% CI 0.71–0.95]; *p* = 0.008),(NNT 14). Comparable results were obtained by analyzing 5-year disease-free survival (RR 0.86 [95% CI 0.76–0.98]; *p* = 0.02 (Figure 5A).

All RCTs [17, 18, 20, 21, 22] analyzed 5-year local control. Adding radiotherapy to chemotherapy favored effect of chemotherapy in all RCTs. An impressive reduction of local recurrence was obtained (RR 0.54 [95% CI 0.40–0.73]; *p* < 0.0001, (NNT 12) No significant benefit was acquired in distant metastasis rate (RR 0.85 [95% CI 0.70–1.05] *p* = 0.13).

### Postoperative radiochemotherapy versus surgery alone

Four randomized trials [14] (15) [16, 4] (773 subjects) analyzed postoperative radiochemotherapy to only surgery. After pooling these studies, no statistically significant gain for 3-year overall survival emerged (RR 0.92 [95% CI 0.82–1.02]; *p* = 0.12) (Figure 2B). A statistically significant difference was confirmed for 3-year disease-free survival pooling data of two RCTs [16, 4]; RR 0.80 [95% CI 0.65–0.98]; *p* = 0.03 (NNT 12) (Figure 4B). For 5-year overall survival, a statistical significant benefit was demonstrated pooling data from three RCTs [4, 15, 16], RR 0.79 [95% CI 0.71–0.87]; *p* < 0.00001 (NNT 6) (Figure 3A) and for 5-year disease free survival RR 0.72 [95% CI 0.63–0.83]; *p* < 0.00001 (NNT 5) (Figure 5B).

### Qualitative results

Sensitivity analysis results for 5-year disease free survival and 5-year overall survival are shown in Table 2. Subgroup analyses were performed separately in relation to publication data (excluding trials published before 1990) and quality score (excluding low quality studies). All homogeneity tests reported no statistical significance: overall effect and confidence intervals resulted unaltered. Furthermore, the difference between 5–year disease-free survival with postoperative radiochemotherapy were comparable by analyzing studies using D2 or studies including a high rate of stages III and IV stages. A subgroup analysis was performed according to the trial's country (eastern vs western countries), no difference in 5-year overall survival was reported.

**Table 2:** Sensitivity analysis

Strata of sensitivity-analysis Results for Each End Point	Subgroup (*n*)	References	RR (CI)	*p*-value
**Exclusion of articles published before 1990**	–	–	–	–
5-yr disease free survival	Article published after 1990	[4] [17] [18] [19] [21] [22]	0.81 (0.72–0.91)	0.0005
5-yr overall survival	Article published after 1990	[4] [17] [18] [19] [21] [22]	0.88 (0.78–1.00)	0.04
**Exclusion of low quality trials**				
5-yr disease free survival	Jadad > 5	[4] [19] [21] [22]	0.78 (0.70–0.86)	< 0.00001
5-yr overall survival	Jadad > 5	[4] [19] [21] [22]	0.85 (0.74–0.98)	0.02
**Exclusion of trials with ≤ 60% of ≥ III stage**				
5-yr disease free survival	>60% of ≥ III stage	[17] [18] [19] [21]	0.87 (0.76–1.01)	0.06
5-yr overall survival	> 60% of ≥ III stage	[17] [18] [19] [21]	0.90 (0.78–1.05)	0.17
Exclusion of trials with ≤ 60% D2 dissection	–	–	–	–
5-yr disease free survival	> 60% D2 dissection	[18] [19] [21] [22]	0.82 (0.72–0.95)	0.007
5-yr overall survival	> 60% D2 dissection	[18] [19] [21] [22]	0.86 (0.74–1.01)	0.06
**Exclusion of Eastern Countries trials**	–	–	–	–
5-yr disease free survival	Western countries	[4] [16] [17]	0.81 (0.62–1.06)	0.13
5-yr overall survival	Western countries	[4] [15] [16] [17]	0.82 (0.74–0.90)	< 0.0001

### Publication bias

The publication bias funnel plot for 5-year overall survival, is presented in Figure 6. This graph shows symmetry suggesting no publication bias.

**Figure 6:** 5-year funnel plot in 5 year overall survival A symmetry in this graph does not indicate publication bias.

## DISCUSSION

The main clinical question of this study is to investigate whether postoperative radiochemotherapy is more efficacious than postoperative chemotherapy or only surgery for increasing the outcome in resected gastric cancer patients. In this literature meta-analysis on 1944 patients in 10 RCTs, we noted an improved 5-year overall survival due to radiotherapy versus postoperative chemotherapy or surgery alone.

The management of gastric carcinoma should be related to the disease's natural history, which is characterized frequently by a local spread. About 50% of patients with advanced gastric cancer will experience a recurrence, of which about 30% will be a local recurrence, even when resection has been considered curative [8]. In this context, radiotherapy has as its rationale to increase local control, especially when delivered with chemotherapy. Confirming all that we have suggested, a significant reduction in the rate of disease control at 3 years and 5 years by radiochemotherapy was observed in all trials but one [17] in which a large difference in patients enrolled in two arms was observed. This advantage is reflected in a gain in overall survival. A significant increase in local control was found in RCTs when comparing postoperative radiochemotherapy versus chemotherapy alone, while no differences were noted in the number of distant metastases. Chemotherapy delivered postoperatively with radiotherapy could conceivably enhance only RT response (radio sensitizer). Indeed, chemotherapy increases the benefit in local control but it does not increase distant metastasis control.

Already in 2001, MacDonald [4] demonstrated a highly significant survival advantage to adjuvant therapy. After a complete resection with negative margins, patients were staged, stratified and subsequently randomized to only surgery or surgery plus adjuvant therapy. The main criticism of this RCT was the inadequate surgical technique with a D0 node dissection. A SEER (Surveillance, Epidemiology, and End Results) analysis of 11630 gastric cancer patients [25] emphasized the role of adjuvant radiotherapy in node-negative patients when less than 15 lymph nodes were removed (HR 1.27, CI 1.08–1.5, *p* = 0.004) and in all patients with positive lymph nodes (5-year overall survival of 30% with adjuvant radiotherapy vs 21% without RT).

The focus clinical point is undoubtedly whether radiotherapy should be added to postoperative chemotherapy, as D2 node dissection had significantly decreased local recurrences. A large observational study analyzed the impact of radiochemotherapy in patients operated with D2 node dissection. [26] This observational study proposed that adjuvant radiochemotherapy in D2-resected gastric-cancer patients could increase overall survival and local control, since a benefit of 6.1% in 5-year overall survival and 6.6% in 5 year disease-free survival was showed in patients treated with radiochemotherapy compared to patients treated surgically only. The same conclusion was reached in a study by Leong [27], in which adjuvant radiochemotherapy was well tolerated with acceptable toxicities and reasonable tumor control regardless of D2 dissection.

In this meta-analysis, the robustness of the results was assessed by sensitivity analyses, excluding the trials on the basis of patient- or study-level covariates. A comparable gain in 5-year disease-free survival was reported, even excluding trials with a proportion of III and IV stages > 80% and trials not using D2 lymphadenectomy, suggesting that these two factors did not influence final results.

Therefore, with the addition a radiotherapy there was a demonstrable benefit of 11% on the 5 year disease-free survival in all RCTs, whereas when analyzing RCTs using only D2 dissection (19, 21, 22) a benefit of 8% was achieved.

This study reports the variations of the outcomes in the different studies not inpatient (we took into consideration the average of the groups rather than individual data). The accuracy of these results could therefore be affected by a lack of other potential confounders. Since this meta-analysis was carried out with summary data, a further meta-analysis of individual patient data to achieve more reliable results would be advisable. We are confident in our accurate manual and computer search retrieval of the published studies including those belonging to non-English literature, and believe that in this study publication bias is not substantial and it is therefore improbable it could alter the results of this pooled analysis.

## MATERIALS AND METHODS

### Selection of randomized trials

This meta-analysis was performed according to the QUOROM statement [9]. Retrieval of randomized controlled trials (RCTs) was based on the Cochrane Controlled Trials Register, The Cochrane Library, MEDLINE, CANCERLIT and EMBASE, limiting the search to randomized clinical trials and human studies and using the following medical subject headings: *gastric carcinoma, radiotherapy, chemotherapy, chemoradiotherapy, randomized trial and clinical trial.* The search included literature published through to December 2016. The computer search was supplemented with manual searches of reference lists for all available review articles, primary studies and bibliographies of books in order to identify other studies not found in the computer search. Abstracts published in the proceedings of the 1999 through 2016 annual meeting of the American Society of Clinical Oncology (ASCO) and the American Society for Therapeutic Radiation and Oncology (ASTRO) were also searched for relevant information. When the results of a single study were reported in more than one publication, only the most recent and complete data were included in the meta-analysis.

### Review of the trials

The RCTs were first reviewed using a list of predefined, pertinent issues that concerned the characteristics of patients and treatments. The quality of each fully published trial was assessed with the Jadad score, using information on study design, method of random assignment, blinding and withdrawal [10]. Total methodological quality scores were then used to rank the studies. Methodological quality assessment was independently performed by two of the authors (F.F., M.M.). Discrepancies among reviewers were infrequent (overall inter-observer variations < 10%), and were resolved by discussion.

### Statistical methods

The crude rates of 3-year and 5-year overall survival were assessed as measures of the treatment's effect. If these data were not available (11) we used the Kaplan-Meier estimates of 5-year overall survival in the treated and control groups reported in the text. When possible, we also analyzed the 3-year and 5-year rates of disease-free survival. Evaluation of therapeutic effectiveness was made with an intention-to-treat method. When not reported in the trial, the response rate according to intention-to-treat was calculated. Differences observed between the two groups were expressed as the pooled relative risk (RR), with its 95% confidence interval (CI). The effect of treatment on the defined outcome measures was calculated from the study data using models based on both fixed and random effects assumptions. In addition to within-study variance, the random effects model considers heterogeneity among studies. Because of the different clinical settings and groups of subjects analyzed, and because the tests for heterogeneity lack statistical power due to the few studies included in this meta-analysis, we have presented the results of random effects models introduced by DerSimonian and Laird [11]. Statistical heterogeneity between trials was evaluated using the Mantel Haenszel χ^2^ test [12]. The number needed to treat (NNT) for benefit which derive from the inverse of the absolute difference of risk among treatment groups, was also used as a measure of the benefits of treatment. We, in turn, excluded each study to ensure that no single study would be solely responsible for the significance of any result of the robust analysis. All our analyses were computed using Revman 5.0. To detect and evaluate clinically significant heterogeneity, we performed several sensitivity analyses in order to identify potential differences in treatment across the studies. First, we estimated whether the type of lymphadenectomy could influence the results of our meta-analysis. The second factor evaluated was the influence of the Jadad quality score (high ≥ 6 or low ≤ 5) of each fully published trial. Thirdly, we performed a sensitivity analysis by excluding those trials that included a high rate of patients at stages I and II. Publication bias was assessed by the Begg and Mazumdar adjusted rank-correlation test for publication bias [13].

## CONCLUSIONS

In patients with resected gastric carcinoma, the available evidence from the literature data is sufficient to conclude the following: 1) the addition of radiotherapy to postoperative chemotherapy improves overall survival; 2) the rate of disease-free survival is significantly influenced by postoperative radiochemotherapy; 3) a gain in 5-year disease- free survival is retained with D2 dissection.
